# Novel preconditioning strategies for enhancing the migratory ability of mesenchymal stem cells in acute kidney injury

**DOI:** 10.1186/s13287-018-0973-3

**Published:** 2018-08-23

**Authors:** Lingfei Zhao, Chenxia Hu, Ping Zhang, Hua Jiang, Jianghua Chen

**Affiliations:** 1 Kidney Disease Center, the First Affiliated Hospital, College of Medicine, Zhejiang University, Hangzhou, Zhejiang People’s Republic of China; 2 Key Laboratory of Kidney Disease Prevention and Control Technology, Hangzhou, Zhejiang Province People’s Republic of China; 3 Institute of Nephrology, Zhejiang University, Hangzhou, Zhejiang People’s Republic of China; 4 State Key Laboratory for Diagnosis and Treatment of Infectious Diseases, the First Affiliated Hospital, College of Medicine, Zhejiang University, Hangzhou, Zhejiang People’s Republic of China

**Keywords:** Mesenchymal stem cells, Migratory ability, Acute kidney injury, Preconditioning strategy

## Abstract

Acute kidney injury (AKI) remains a worldwide public health issue due to its increasing incidence, significant mortality, and lack of specific target-orientated therapy. Developments in mesenchymal stem cell (MSC) research make MSCs a promising candidate for AKI management but relevant clinical trials show confusing results (NCT00733876, NCT01602328). One primary cause of the limited therapeutic effect may result from poor engraftment of transplanted cells. To solve this problem, investigators have developed a series of preconditioning strategies to improve MSC engraftment in animal AKI models. In this review, we summarize these previous studies, providing an integrated and updated view of different preconditioning strategies aimed at promoting the therapeutic effect of MSCs in AKI patients.

## Background

Acute kidney injury (AKI) is a common clinical disease defined as an abrupt decline in glomerular filtration, resulting in dysregulation of extracellular volume and electrolytes, which can subsequently induce a series of complications and failure of other organs [1]. The causes of AKI are numerous, including renal ischemia, nephrotoxins, sepsis, and so on. Although much work has been completed in this area over recent decades, the prevalence of AKI is still rapidly increasing [2, 3]. It is estimated that the worldwide occurrence of AKI has reached approximately 13 million people per year. For inpatients, 5% of all hospitalized patients and 40% of critically ill patients may develop AKI during their hospitalization [4, 5]. Except for the high morbidity rate, the prognosis of AKI is also not very good. The mortality rates in intensive care unit patients with AKI can reach 50–70% [6] and those who survive the acute phase also bear a high risk of developing chronic kidney disease (CKD). A recent meta-analysis found an 8.8-fold increase in risk for CKD and a 3.3-fold increased risk for end-stage renal disease (ESRD) in patients surviving AKI after hospital discharge [7]. Both the high morbidity rate and poor prognosis place a heavy burden on the public health care system, as it is estimated that the annual medical expenses for AKI treatment have exceeded $10 billion in the US and £400–600 million in the UK [8].

Currently, therapeutic choices are still confined to supportive care and preventive strategies, since kidneys have a remarkable self-repair capacity [9]. However, none of these appear to have decreased the mortality rate [10]. Some drugs have also been explored for preventing or treating AKI, such as diuretics, dopamine, fenoldopam, atrial natriuretic peptide, recombinant human insulin-like growth factor-1 (IGF-1), and erythropoietin (EPO) [11–15]. Despite good results in animal experiments, there is still limited evidence for their use in humans according to KDIGO-AKI guidelines [16]. During the past decade, we have witnessed an explosion of cell-based therapy in clinical use. While pharmacologic interventions often target only a single aspect of the highly complex pathophysiology following AKI, cell-based therapies may have the advantage of acting through multiple mechanisms to promote tubular epithelial cell repair [17]. Thus far, according to ClinicalTrials.gov, more than 4000 clinical trials employing stem cells from different origins have been conducted, and 46 of those consist of mesenchymal stem cell (MSC) therapy for AKI and CKD [18–22]. Application of MSC therapy may become a potentially effective supplemental regimen for current situations.

## MSC therapy and its application in AKI

MSCs are fibroblast-like multi-potent cells first identified by Friedenstein in the 1960s and 1970s [23]. They are characterized by the robust ability for self-renewal, regeneration, proliferation, and multi-lineage differentiation [24]. By exposure to appropriate conditions, MSCs can differentiate into adipocytes, chondrocytes, and osteocytes [25]. MSCs were initially isolated from bone marrow, but now various sources, including placenta, amniotic fluid, umbilical cord blood, Wharton’s jelly, and adipose tissue, are available for preclinical and clinical use [26]. Due to very high variability in MSC preparations [27], in 2006 the International Society of Cell Therapy (ISCT) proposed criteria for the definition of MSCs: adherence to plastic with the capacity to differentiate into chondrocytes, osteoblasts, and adipocytes in in vitro culture conditions; positive for CD105, CD73, and CD90; negative for the hematopoietic markers CD45, CD34, CD19, CD79 and HLA-DR expression on the cell surface [28].

MSCs secrete a number of factors, including transforming growth factor-β (TGF-β), hepatocyte growth factor (HGF), vascular endothelial growth factor (vEGF), and IGF-1, which can exert anti-apoptotic [29, 30], immunomodulation [31, 32], anti-oxidative [33, 34], and pro-angiogenic factors [35, 36] and target almost all pathophysiological components of AKI. MSCs can also release plenty of microvesicles (MVs), which are particularly enriched in specific molecules, especially functional mRNAs and microRNAs. Their role in vivo may be related to cell-to-cell communication and to protein and RNA exchange among cells both locally and at a distance [37]. In addition to their paracrine/endocrine activity, some studies have also demonstrated MSCs may have the ability to directly differentiate into target cells [38, 39]. This point has not been accepted by all experts, however, because most MSCs may disappear from the kidney and other organs within 72 h after infusion, which is not enough time for differentiation [40, 41] (Fig. 1).

**Fig. 1:** Renal repair function of MSCs in acute kidney injury. After infusion, MSCs temporarily adhere to glomerular and postglomerular capillaries. Through a series of mechanisms, MSCs exert anti-apoptotic/anti-oxidative, anti-inflammation, immunomodulation, and pro-angiogenic effects. **a** Cytokines and growth factors are delivered to the injured tubular cells through paracrine actions. **b** This mechanism can also proceed through endocrine actions. **c** MSCs can secrete plenty of microvesicles, which are particularly enriched in functional mRNAs and microRNAs. Crosstalk between microvesicles and injured tubular cells causes beneficial changes in the respective gene expression profiles. **d** Some studies have also demonstrated MSCs may have the ability to directly differentiate into target cells

Adequate evidence demonstrates that MSCs are effective in improving outcome after AKI in different animal models. The majority of animal models included are cisplatin-induced AKI, sepsis-associated AKI, ischemia-reperfusion injury, and glycerol-induced AKI, covering most causes of human AKI [41–46].

Besides the excellent outcomes in animal models, two clinical trials have been explored on the use of MSCs in the AKI setting, but results remain contradictory. In a 2008 phase I clinical trial (NCT00733876), the safety and efficacy of MSCs were demonstrated in patients who were at high risk (underlying CKD, advanced age, diabetes mellitus, congestive heart failure, chronic obstructive lung disease, and prolonged pump times) of developing AKI after undergoing on-pump cardiac surgery. After analyzing data from 18 included patients, they concluded MSCs were useful for protecting against AKI development (0% AKI incidence in MSCs group versus 20% in control group) [47]. Based on this positive result, another phase II, randomized, double-blind, multicenter trial used MSCs to treat patients for postcardiac surgical AKI (NCT01602328) in 2017 [48]. They randomized 156 adult subjects and, at the end of the study, time to renal function recovery, the need for dialysis, and 30-day all-cause mortality were compatible between MSCs group and control group. These contradictory results are confusing to physicians when treating AKI patients because of the high price and potential tumorigenicity of MSC therapy. We need more clinical trials to address these issues, and another ongoing trial (NCT03015623) may give us clear insight into the role of MSC therapy for AKI patients (Table 1).

**Table 1:** Clinical trials on MSC application in AKI

Aim of study	Enrollment	Phase	Status	ClinicalTrials.gov identifier
To determine if the administration of allogeneic MSCs at defined doses is safe in patients who are at high risk of developing significant AKI after undergoing on-pump cardiac surgery	18	Phase I	Completed	NCT00733876
To determine the safety and efficacy of allogeneic human MSCs in reducing the time to recover from AKI after cardiac surgery	156	Phase II	Terminated	NCT01602328
To assess the safety and tolerability of SBI-101, a biologic/device combination product using allogeneic human MSCs in subjects with AKI	24	Phase I	Recruiting	NCT03015623

*AKI* acute kidney injury, *MSC* mesenchymal stem cell

## Concerns about the clinical application of MSCs in AKI

Some concerns remain regarding the clinical application of MSCs in AKI. First, considering their antigenicity, previous studies were performed using autologous MSCs to avoid immune rejection of donor cells [49]. However, the high expense, complex process, and timing constraints of the harvesting period from individual patients restricts their application clinically. What is more, autologous MSCs obtained from elderly donors and those with multiple medical comorbidities have significantly reduced capacity for proliferation and differentiation, with increased apoptosis signals hampering their use in the patients who will get the most benefit from such therapy [50, 51]. In fact, the absence of major histocompatibility class II antigens (MHC II) makes MSCs immunoprivileged in vivo, and increasing experimental findings have suggested autologous MSC therapy has comparable safety and effectiveness in both the short and long term after AKI [44, 52]. According to a mapping and multiscale analysis in 2016, the number of registered trials using allogeneic MSCs exceeded those with autologous MSCs (53% versus 47%) [53].

The second concern is the precise definition of MSCs. The criteria proposed by ISCT in 2006 is a minimum standard for identifying MSCs. MSCs from various sources, however, may have different biological characteristics [54–57]. Recent studies on pericytes even challenge the widely accepted view of endogenous pericytes as MSCs and suggest their progenitor potential is induced by artificial conditions and high concentrations of mitogens ex vivo [58]. This evidence raises the concern that the current definition of MSCs, which is based on surface markers and/or differentiation parameters, may not be the optimum criteria for MSCs. However, using specific DNA methylation patterns has bright prospects with regard to MSC classification [59]. In 2017, a concise review suggested using multiple methods, such as genomic, epigenomic, transcriptomic, proteomic, and metabolomic, to measure colony-forming ability, CD marker expression, telomere length, and cellular morphology, which may be useful to establish a next-generation definition for MSCs [60].

The required dose of MSCs for clinical therapy and its relevance to injury repair is a topic of active research. Although there is still no related clinical data for AKI, a preclinical study suggests medium-dose and high-dose MSC therapy (2 × 10^6^ and 5 × 10^6^ MSCs per kilogram bodyweight) result in better renoprotective effects after AKI compared with low-dose therapy [44]. Data from another phase I/II multicenter randomized controlled clinical study for the treatment of knee osteoarthritis also confirmed this dose-related effect [61]. This relationship may be more complicated in the field of cardiac regeneration as some are demonstrating a direct and others an inverse dose response [62–65]. It seems that different tissues need different doses of MSC therapy for repair, and more large population and appropriate control studies in the future may help us to obtain a more definitive answer to this question.

Finally, why do relevant clinical trials in AKI show confusing results? One explanation for the limited effect of MSC therapy in human AKI may be the relatively low number of transplanted MSCs in kidneys. MSCs either die due to the harsh microenvironment in vivo or cannot find their way to the injured kidneys [66, 67]. Only 1% of the delivered cells reach the target site, while most are trapped in the liver, lungs, and spleen [68–72]. Investigators have attempted to increase the number of injected cells but this may be risky as disturbances in blood flow may cause embolism problems [73]. Others have attempted to inject cells into the damaged tissue directly, but the invasive procedures include a high risk of hemorrhage and the number of injected MSCs is also not accurate because most of the cells may escape from the injected site [74, 75]. To strengthen the therapeutic potential of transplanted MSCs, many innovative preconditioning methods have been explored and shown excellent results in recent years [76, 77]. Below, we will discuss these novel strategies.

## Preconditioning can enhance the migratory ability of MSCs

Based on the way MSCs work, these strategies are designed to either increase the effective quantity of MSCs in injured tissues (e.g., increase the survival rate of MSCs or promote their homing ability) or enhance their paracrine/endocrine ability (Fig. 2). Of these, improvement of MSC homing is of great importance because there is evidence that culture-expanded MSCs may lose a few surface molecules and be unable to migrate [67, 78, 79]. Understanding the MSC homing mechanisms may help us solve this problem.

**Fig. 2:** Once injected in vivo, MSCs face a harsh microenvironment that may induce their senescence or apoptosis. Different preconditioning methods like hypoxia, gene modification, cytokines, etc. are key strategies to improve MSC function in tissue repair. *ROS* reactive oxygen species

After an injury, chemokines are released by the injured organ. By chemotaxis, MSCs can follow the gradient of soluble chemoattractants to the injured site. Then, with the help of sequences of molecular and cellular events, MSCs experience rolling and adhesion and finally transmigrate across the endothelium [80–86]. Based on this theory, some novel preconditioning strategies being explored either increase the affinity of MSCs to migratory stimuli or modulate the target sites to secrete more chemokines.

### Increasing the affinity bility of MSCs to migratory stimuli (MSC-based strategies)

MSCs express many chemokine receptors on their surface which play an essential role in their migration by interaction with appropriate ligands. Currently, over 50 chemokines and 20 chemokine receptors have been discovered [87]. According to their cysteine residues, they have been divided into four categories: CXC family, CC family, XC family, and CX3C family [88]. Different isolation techniques and in vitro culture conditions may change the MSC expression of chemokine receptors [89, 90], but it has been widely acknowledged that CCR1, CCR2, CCR7, CXCR4, CX3CR1, CXCR6, c-met, and CD44 are primarily linked to the in vivo migratory abilities of MSCs [91–93].

The stromal derived factor-1 (SDF-1)/chemokine (C-X-C motif) receptor 4 (CXCR4) axis plays an important role in governing stem cell homing and engraftment in the bone marrow following transplantation [94–96]. SDF-1 is a member of the chemokine family and is widely expressed by both bone marrow-derived mesenchymal stromal cells (BMSCs) and endothelial cells [94] and is predominantly promoted under ischemic conditions, including AKI [97–99]. CXCR4, which can act as its unique receptor, is expressed on human stem and progenitor cells [100]. Unlike the abundant CXCR4 expression on hematopoietic stem cells, only approximately 1% of all human BMSCs present CXCR4, and most of the CXCR4 mRNA and antigen (83–98%) is expressed inside cells [101, 102]. Furthermore, after four to five passages of ex vivo expansion, its expression becomes barely detectable, which largely decreases the homing ability of the cells [103, 104]. Multiple strategies, such as incubation with cytokines or chemical compounds, co-injection, hypoxia stimulation, and genetic modifications, have been explored as novel preconditioning methods to enhance the interaction of SDF-1 with CXCR4 (Table 2).

**Table 2:** Different preconditioning methods to enhance the interaction of SDF-1 with CXCR4 in AKI models

Year	Animal	AKI model	MSC source	Preconditioning	Outcomes	References
2012	Rat	I/R	BM	Incubation with cytokines or chemical compounds	Increased SDF-1 level, migration, survival, secretory capacity	[10]
2013	Mice	Cisplatin	BM	Incubation with cytokines or chemical compounds	Increased CXCR4 expression, migration, survival, secretory capacity	[105]
2014	Rat	Gentamicin	BM	Co-injection	Increased CXCR4 and CXCR7 expression, migration, proliferative ability, secretory capacity	[108]
2013	Mice	I/R	BM	Co-injection	Increased SDF-1 level, migration	[109]
2013	Rat	I/R	BM	Hypoxia stimulation	Increased HIF-1α and CXCR4 expression, migration, retention time, secretory capacity	[114]
2013	Rat	I/R	BM	Genetic modification	Increased CXCR4 expression, migration, secretory capacity	[115]

*AKI* acute kidney injury, *MSC* mesenchymal stem cell, *I/R* ischemia/reperfusion, *BM* bone marrow, *SDF-1* stromal-derived factor-1, *CXCR* chemokine (C-X-C motif) receptor, *HIF* hypoxia-inducible factor

#### Incubation with cytokines or chemical compounds

Incubation with cytokines or chemical compounds is a simple and fast preconditioning strategy for MSCs. Some cytokines or chemical compounds can trigger signaling pathways, leading to the overexpression of CXCR4. After preconditioning with 20 ng/ml IGF-1 for 24 h, MSCs were transplanted into a cisplatin-induced AKI mice model [105]. This method successfully resulted in increased cell survival rate and robust migration of MSCs towards the ischemic site followed by structural and functional recovery. This phenomenon was caused by a twofold increase in CXCR4 expression on the MSC surface [105]. Pretreatment with S-nitroso N-acetyl penicillamine, which serves as a nitric oxide donor, caused transplanted MSCs to significantly up-regulate the level of SDF-1, which resulted in better survival and migratory and secretory ability [10].

#### Co-injection

A synergistic effect is common in pharmacology and co-injection with drugs can enhance the migratory ability of MSCs. Muscone is the main active ingredient of musk with a supposed function as a refreshing agent, promoting blood flow and detumescence [106, 107]. Preconditioning with muscone significantly improved BMSC engraftment in injured kidney as well as other bioactivities, including cell proliferation and secretion, with increased expression of both CXCR4 and CXCR7 in gentamicin-induced AKI rats [108]. Pretreatment with EPO significantly increased this chemotactic effect of transplanted MSCs in an ischemia/reperfusion-AKI (IR-AKI) model, because EPO can increase SDF-1 levels in the AKI microenvironment and activate the PI3K/AKT and MAPK signaling pathways in MSCs [109].

#### Hypoxia

The low oxygen tension in injured organs may become another obstacle for the application of MSCs which are cultured under normal oxygen tension. Once localized to the ischemic tissue, MSCs encounter more severe hypoxic conditions, ranging from 0.4 to 2.3% O_2_, which often results in apoptosis [110]. Pre-exposure of MSCs to hypoxia may activate the expression of some genes, e.g., those encoding CXCR4, CXCR7, CX3CR1, SDF-1α, and hypoxia-inducible factor (HIF), all of which take part in cell migration [111–113]. In addition, cobalt is a kind of hypoxia mimetic preconditioning agent which significantly enhances MSC migratory ability by activating HIF-1α and up-regulating CXCR4, promoting improved morphology and function following AKI [114].

#### Genetic modifications

Genetic modifications which make MSCs overexpress migratory genes is a more accurate way to enhance MSCs’ migratory ability compared with other preconditioning strategies. For example, overexpression of CXCR4 in BMSCs effectively promoted the migration of BMSCs to the injured site of the kidney by their paracrine actions, resulting in greater improvement in renal function [115]. However, the effect was entirely abolished by pre-incubation with AMD3100, a CXCR4-specific antagonist, further confirming the important role of the SDF-1/CXCR4 axis in MSC migration [115].

#### Next-generation preconditioning strategies

With the development of bioengineering, some novel preconditioning approaches are being explored, such as the use of hydrogels or microgels. Using MSC engineering with biomaterials could mimic cellular microenvironments more consistent with those encountered in vivo and deliver more cells to injured tissues. Although the mechanism has not been clarified, improvement of cell engraftment was observed while using an IGF-1C domain-modified chitosan hydrogel in IR-AKI model rats, which suggests enhanced MSC migratory ability through hydrogel delivery [116]. Similarly, a spherical, naturally derived extracellular matrix-based, type-I collagen microgel led to MSCs expressing significantly increased levels of SDF-1 and offered a significant functional improvement in a hind-limb ischemia mouse model [117].

### Modulating target site secretion of chemokines (site-based strategies)

Apart from various methods focusing on improving the migratory function of MSCs, stimulation of the host tissue to promote recruitment is another feasible strategy. Magnification of the naturally occurring electric fields at sites of bone fracture may become a powerful cue in directing migration of human MSCs [118]. Pulse-focused ultrasound (pFUS) has been shown to enhance the homing of human MSCs through mechanotransduction, eliciting transient local increases of chemoattractants in healthy murine skeletal muscle and kidneys [119, 120]. Recently, Burks et al. [121] targeted pFUS to kidneys of mice suffering from cisplatin-induced AKI in order to evaluate whether this method could enhance MSC homing and relieve renal injury. Following pFUS treatment, tissue levels of many known chemoattractants were significantly altered, and the pFUS+MSC group had more MSCs home to the kidney and better renal function compared with the MSC group. They demonstrated pFUS could be a neoadjuvant approach to improve MSC homing to diseased organs.

## Conclusions

Despite encouraging results in animal models, a large gap between scientific observation and clinical application of MSCs still exists. Improvement of MSC homing is a major challenge in clinical applications. Several preconditioning strategies have been established for enhancing the migratory ability of MSCs in AKI models. In our review, we summarize these studies and conclude that the improvement of migratory effects are mostly through the SDF-1/CXCR4 axis.

Some concerns should also be considered when applying these preconditioning strategies. Genetic modification methods are thought to have potential tumor progression risk, but so far no tumorigenic transformational changes have been observed. For pFUS, tissue damage following stimulation needs to be carefully monitored, especially using pFUS with microbubble ultrasound contrast agents. As well as the strategies discussed, investigators have also explored many other preconditioning agents, such as equipped scaffolds, melatonin, MSC-derived MV, and so on. In our opinion, combination of MSC-based and target site-based strategies may further improve the therapeutic effects and lead to better subsequent outcomes.

Another important issue for MSC application in AKI is the need for potency assays. Due to the heterogeneous population of cells and multiple mechanisms of action, no consensus on a potency assay for MSCs has been achieved. Considering their complex biological qualities, an assay matrix using biologic assays, biologic and analytical assays, or analytical assays alone to assay anti-apoptotic, immunomodulation, anti-oxidative, pro-angiogenic, and migratory functionalities of MSCs may be a proper tool to verify a specific intended effect between different MSC products and expand their application clinically.

To this end, we look forward to an optimistic future of cell-based therapy in kidney disease, while understanding the pathophysiology of AKI and clarifying the renoprotective mechanism of MSCs may further expand the success of regenerative medicine using MSCs for treating AKI.

## Abbreviations

AKI: Acute kidney injury
BMSCs: Bone marrow-derived mesenchymal stromal cells
CKD: Chronic kidney disease
CXCR4: Chemokine (C-X-C motif) receptor 4
EPO: Erythropoietin
ESRD: End-stage renal disease
HGF: Hepatocyte growth factor
HIF: Hypoxia-inducible factor
IGF-1: Insulin-like growth factor-1
IR-AKI: Ischemia/reperfusion-AKI
ISCT: International Society of Cell Therapy
MHC II: Major histocompatibility class II
MSCs: Mesenchymal stem cells
MV: Microvesicles
pFUS: Pulse-focused ultrasound
SDF-1: Stromal derived factor-1
TGF-β: Transforming growth factor-β
vEGF: Vascular endothelial growth factor
